The article "Unilateral Multifocality and Bilaterality Could Be Two Different Multifocal Entities in Patients with Papillary Thyroid Microcarcinoma" was retracted in 2024. Reasons: signs of a paper mill; suspected computer-generated content; unreliable results or conclusions; concerns about the data.

# Unilateral Multifocality and Bilaterality Could Be Two Different Multifocal Entities in Patients with Papillary Thyroid Microcarcinoma

**DOI:** 10.1155/2020/9854964

**Published:** 2020-07-03

**Authors:** Junbo Cai, Fang Fang, Jianbin Chen, Dapeng Xiang

**Affiliations:** ^1^Department of General Surgery, Taizhou Municipal Hospital, Taizhou, Zhejiang, China; ^2^Department of General Surgery, The Second Affiliated Hospital of Zhejiang University, School of Medicine, Hangzhou, Zhejiang, China

## Abstract

**Objective:**

Multifocality within an affected lobe (unilateral multifocality) or two lobes (bilaterality) is commonly denoted as multifocality without differentiation. Recently, there has been molecular evidence indicating that unilateral multifocality and bilaterality could be two different entities. However, few studies concerning the comparison between these two different multifocality entities have been reported.

**Design:**

A retrospective cohort study.

**Methods:**

From 2010 to 2013, in total, 949 consecutive patients with papillary thyroid microcarcinoma (PTMC) were enrolled and further divided into four groups based on multifocality status. Unilateral multifocality and bilaterality were analyzed by binary logistic regression along with other clinicopathological factors.

**Results:**

Unilateral multifocality, instead of bilaterality, was correlated with central neck metastasis (CNM) in both univariate and multivariate analyses. Group IV (unilateral multifocality and bilaterality coexist) had the highest CNM rate. Group III (unilateral multifocality) had a higher CNM rate than group II (bilaterality, single lesion in each lobe), with a significant difference (*p* = 0.032). Similar lateral neck metastasis tendency was observed among the four groups. In the multivariate analysis, only unilateral multifocality and bilaterality which coexisted were correlated with CNM. Moreover, 9 cases had a recurrence, with the recurrence rate ranking top in group IV (3.6%), second in group III (2.8%), and third in group II (1.2%). The difference was significant (*p* = 0.021).

**Conclusion:**

Unilateral multifocality and bilaterality could be two different multifocal entities in patients with PTMC. Unilateral multifocality serving as a prognostic factor indicated a worse prognosis than bilaterality on neck metastasis. When the two factors coexisted in PTMC, patients had the highest risk of CNM and possibly local recurrence compared with those with either risk factor alone.

## 1. Introduction

Papillary thyroid microcarcinoma (PTMC) is a papillary thyroid carcinoma (PTC) less than 10 mm frequently associated with central neck metastasis (CNM). Over the past 3 decades, there has been an increasing incidence of PTMC worldwide [1]. Although the overall prognosis of PTMC is excellent, local recurrence is not rare and some cases even have distant metastasis with lethal consequences [2–7].

The article "Unilateral Multifocality and Bilaterality Could Be Two Different Multifocal Entities in Patients with Papillary Thyroid Microcarcinoma" was retracted in 2024. Reasons: signs of a paper mill; suspected computer-generated content; unreliable results or conclusions; concerns about the data.

The presence of multifocality is a known factor indicating the poor prognosis of PTMC [8]. Increasing lines of studies have found that multifocality is correlated to occult and macroscopic CNM [2, 9–11]. Several large group studies with a long-time follow-up show that multifocality is correlated to local and distant recurrence in PTC [2, 5, 12–15], although some found that there is no significant association [7, 16] Multifocality is defined as two or more carcinoma lesions within the thyroid. Multifocality develops in two kinds of forms: multifocality within one single lobe (unilateral multifocality) or multifocality within two lobes (bilaterality). There is still a controversy with respect to the origin of separate foci in patients with PTC. Some believe that multifocality originates from the same clone and is caused by intrathyroid metastasis, while others argue the opposite [17, 18]. BRAF^V600E^ mutation is the dominant type in sporadic PTCs besides RAS and RET/PTC. They act upon the same linear oncogenic signaling cascade and are mutually exclusive in PTCs [19–21]. Under this premise, Bansal et al. recently have found that multifocality mostly originates from different mutations, and unilateral multifocality tends to share the same mutation while bilaterality generally has a different mutation status [22]. This study partially provides molecular evidence that unilateral multifocality and bilaterality could be two different kinds of multifocal entities.

There have been many reports trying to reveal the prognostic value of multifocality in patients with PTC. However, most of previous studies did not separate unilateral multifocality from bilaterality, and they are commonly denoted as multifocality without differentiation. We supposed that unilateral multifocality and bilaterality are two different kinds of entities with different biological and clinical characteristics leading to different outcomes. To better investigate the prognostic value of these two kinds of multifocality, we conducted this retrospective study based on a large series of PTMC patients.

## 2. Subjects and Methods

### 2.1. Patients

The study design and protocol were approved by the Ethics Committee of Second Affiliated Hospital, Zhejiang University College of Medicine. From May 2010 to January 2013, medical records of 1,156 consecutive patients with PTMC were reviewed for patient demographic, clinical and radiological examination results, operative procedure, and pathological examination result. 949 patients with PTMC were finally enrolled. The patients included in the study met the following criteria: all patients had papillary thyroid tumor of 1.0 cm or less in diameter by final pathological examination and no previous thyroid surgery or an adequate medical history. Incidental PTMCs found during operation or after thyroidectomy without neck dissection were excluded.

The article "Unilateral Multifocality and Bilaterality Could Be Two Different Multifocal Entities in Patients with Papillary Thyroid Microcarcinoma" was retracted in 2024. Reasons: signs of a paper mill; suspected computer-generated content; unreliable results or conclusions; concerns about the data.

### 2.2. Assessment of Clinicopathological Variables

The following variables were analyzed as risk factors for neck metastasis: unilateral multifocality (multifocal tumors within one lobe), bilaterality (lesions at both lobes), gender, age at diagnosis (<45 yrs vs. ≥45 yrs), maximal tumor size (the largest dominant tumor size for multifocal lesions, ≤0.5 vs. >0.5 cm), capsular invasion, extrathyroidal invasion, intraglandular dissemination, and the concomitant Hashimoto disease or simple goiter. Multifocal lesions were defined as two or more cancer sites within the thyroid and were confirmed by a final pathological examination. Capsular invasion was defined as minimal extrathyroidal extension of the capsule (T3). Extrathyroidal invasion was defined as the extension beyond the thyroid capsule invading subcutaneous soft tissues, the esophagus, or the recurrent laryngeal nerve (T4) [23]. Intraglandular dissemination was defined as the islands of papillary carcinoma cells located at least 500 *μ*m apart from the primary tumor [24].

### 2.3. Surgical Procedures

Total thyroidectomy was performed when the lesions were multifocal in both thyroid lobes. Subtotal thyroidectomy was performed under two conditions: (1) multiple benign nodules were detected at the contralateral lobe and (2) lesions were located at the isthmus. Lobectomy plus isthmus was performed when lesions were limited in a single lobe.

Prophylactic lateral neck dissection (LND) was performed for all enrolled patients. LND was performed cranially to both superior thyroid arteries and the pyramidal lobe, caudally to the innominate vein, laterally to the carotid sheaths, and dorsally to the prevertebral fascia. The ipsilateral central compartment was defined as the prelaryngeal/pretracheal and paratracheal regions ipsilateral to the tumor location. Bilateral LND was performed when lesions were multifocal or located at the isthmus. Selective ipsilateral LND was performed when lesions were confined in one lobe. Selective LND, including Levels II to IV, was performed when suspicious lymph nodes were detected at the lateral neck by imaging examinations or palpation.

### 2.4. Follow-Up

All patients received TSH-suppressive hormonal therapy after surgery and were followed-up every three to six months. US examination, laboratory examination, and laryngoscope were performed at the surgeon's discretion. Locoregional recurrence was detected by US or CT and was confirmed by a cytological examination.

The article "Unilateral Multifocality and Bilaterality Could Be Two Different Multifocal Entities in Patients with Papillary Thyroid Microcarcinoma" was retracted in 2024. Reasons: signs of a paper mill; suspected computer-generated content; unreliable results or conclusions; concerns about the data.

### 2.5. Statistics

The statistical analyses in this study were performed using a statistical package (SPSS 17.0, Chicago, IL). Frequencies were compared using Pearson's chi-square test or Fisher's exact probability test. Univariate analyses of correlations between CNM/LNM (lateral neck metastasis) and clinicopathological variables were performed using Pearson's chi-square test or Fisher's exact probability test. Variables with a *p* < 0.05 in univariate analysis were included in the multivariate analysis with binary logistic regression. In all cases, a *p* value less than 0.05 was considered statistically significant.

## 3. Results

### 3.1. Patients and Clinicopathological Features

From May 2010 to January 2013, medical records of 1,156 consecutive patients with PTMC were reviewed and 949 patients meeting the inclusive criteria were finally enrolled. There were 207 male (21.8%) and 742 female (78.2%) patients with a mean age of 43.8 years (range 16-79). Multifocality was present in 236 patients, including bilaterality in 164 cases and unilateral multifocality in 155 cases. CNM was found in 299 (31.5%) patients, while LNM was present in 44 patients (4.6%) (Table 1). All the 44 patients had suspicious enlarged LNs at the lateral neck, and therapeutic LND from Level II to Level IV was performed. No patient had a family history of thyroid cancer or an exposure history of radiation.

### 3.2. Clinicopathological Factors for CNM and LNM

In univariate analysis, CNM was significantly correlated with unilateral multifocality, age < 45 yrs, male, tumor size > 0.5 cm, capsular invasion, and extrathyroidal invasion. All factors above were included in multivariate analysis. In the multivariate analysis, CNM was significantly correlated with age < 45 yrs, male, tumor size > 0.5 cm, extrathyroidal invasion, and unilateral multifocality (Table 2). The results indicated that unilateral multifocality is a risk factor for CNM.

In univariate analysis, LNM was significantly correlated with male, tumor size > 0.5 cm, and CNM. All factors above were included in the multivariate analysis. In multivariate analysis, tumor size > 0.5 cm and CNM were verified to be correlated with LNM (Table 3).

### 3.3. Correlations between Different Kinds of Multifocality Forms, Neck Metastasis, and Recurrence

Based on multifocality forms, patients were classified into four groups: I—single lesion (*n* = 713), II—bilaterality without multifocality in each lobe (single lesion within each lobe, *n* = 81), III—unilateral multifocality (*n* = 72), and IV—unilateral multifocality and bilaterality coexist (*n* = 83). Four groups were not different regarding age, gender, capsular invasion, extrathyroidal invasion, and Hashimoto. Group II showed the highest proportion of patients with a large tumor size (>0.5 cm), and group III showed the highest proportion of patients with simple goiter (Table 4). Group IV had the highest risk of CNM, with group III being the second and group II being the third. The difference was significant among the four groups (*p* = 0.032). As to LNM, group IV had the highest risk, with group III being the second and group I being the third. The difference was not significant (*p* = 0.266). Similar tendency as CNM was observed on recurrence, and group IV had the highest risk with group III being the second and group II being the third. The difference was significant among the four groups (*p* = 0.021). In the multivariate analysis, unilateral multifocality and bilaterality coexisted (group IV) which was independently correlated with CNM with an OR of 1.823, as well as other strong factors like age < 45 yrs, male, tumor size > 0.5 cm, and extrathyroidal invasion. Univocal bilaterality (group II) and unilateral multifocality (group III) were not correlated with CNM in both univariate and multivariate analyses (Table 5).

The article "Unilateral Multifocality and Bilaterality Could Be Two Different Multifocal Entities in Patients with Papillary Thyroid Microcarcinoma" was retracted in 2024. Reasons: signs of a paper mill; suspected computer-generated content; unreliable results or conclusions; concerns about the data.

These results showed that unilateral multifocality and bilaterality could be two different kinds of entities in patients with PTMC. The comparison between group II and III clearly showed that univocal bilaterality alone did not increase the risk of CNM and recurrence. On the contrary, unilateral multifocality was a strong risk factor for both CNM and recurrence.

### 3.4. Complications and Recurrence

96 patients (10.1%) had transient hypoparathyroidism, and 1 patient (0.1%) had permanent hypoparathyroidism. 31 patients (3%) had temporary vocal cord palsy (recovered within 6 months), and 2 patients (0.2%) had permanent recurrent laryngeal nerve injury. One of the two patients had recurrent laryngeal nerve invasion by tumor, and complete resection of recurrent laryngeal nerve was performed.

The mean length of follow-up was 32.2 months, ranging from 18 to 50 months. During the follow-up period, 9 patients (0.9%) had locoregional recurrence. No patient demonstrated distant metastasis or died.

## 4. Discussion

Multifocality is a commonly seen status, and up to 80% of PTC patients develop multiple tumor foci in the same or both thyroid lobes [25–28]. It remains controversial whether these multifocal PTCs are multiple synchronous primary tumors (MSPTs) arising from independent clones or whether they are the result of intraglandular dissemination of a single malignant clone [18, 22].

The article "Unilateral Multifocality and Bilaterality Could Be Two Different Multifocal Entities in Patients with Papillary Thyroid Microcarcinoma" was retracted in 2024. Reasons: signs of a paper mill; suspected computer-generated content; unreliable results or conclusions; concerns about the data.

Multifocality in PTC was once thought to be caused by lymphatic dissemination of tumor cells from one malignant clone, which is supported by a common finding of tumor cells in the lymphatic vessels and frequent lymph node metastasis. Recently, several studies have tried to address this issue from a molecular prospect. By analyzing microsatellite alterations and X-chromosome inactivation status in 22 multifocal PTC patients, McCarthy et al. conclude that multifocal tumors in PTC patients often arise from the same clone and intrathyroid metastasis may play an important role in the spread of malignancy, while Shattuck et al. argue the opposite finding using approximately the same technique. Most recently, Bansal and colleagues analyzed the molecular characteristics (BRAF, RAS, and RET) and histopathologic status of 60 multifocal PTC patients and found that multifocality in as many as 60% of multifocal PTCs may arise from different origins and they typically located in different lobes. Meanwhile, multifocality within the same lobe tends to share the same mutation status^22^. These findings elucidate that unilateral multifocality is different from bilaterality.

We tried to address this issue on the clinical level in two ways. Firstly, multifocality was separately denoted in two ways and analyzed as two independent risk factors: (a) present with unilateral multifocality or not and (b) present with bilaterality or not. In the present study, 155 (16.3%) patients had unilateral multifocality while 164 (17.3%) patients had bilaterality. In the univariate analysis, unilateral multifocality, instead of bilaterality, was significantly correlated with CNM. In the multivariate analysis, unilateral multifocality was analyzed with other strong factors like tumor size, age, and gender, and it still showed as an independent predictor of CNM with an OR of 1.661 (*p* = 0.008) (Table 2). These results showed that unilateral multifocality is a much stronger risk factor than bilaterality, which partially supports that unilateral multifocality and bilaterality are two different kinds of multifocal entities.

The four groups in this study were largely the same on several analyzed factors except that group II had a significantly higher proportion of tumors > 0.5 cm. We found that group III showed a higher CNM rate than group II (38.9% vs. 32.1%), which was consistent with preliminary analysis. Moreover, group IV showed the highest CNM rate and that of group I was the lowest. The difference was significant among the four groups (*p* = 0.032). Concerning the LNM rate, similar tendency was observed among the four groups although the difference was not statistically significant (Table 4). In the multivariate analysis, only group IV (unilateral multifocality and bilaterality coexist) was independently correlated with CNM. These data showed more precisely that PTMC patients with unilateral multifocality were more prone to have CNM compared with those with univocal bilaterality (single lesion within each lobe). Moreover, when these two factors coexisted, patients showed the highest CNM rate. It is conceivable that when the two risk factors occurred synchronously, the risk of neck metastasis could increase and patients with PTMC are more likely to have CNM than those with either single risk factor alone.

The article "Unilateral Multifocality and Bilaterality Could Be Two Different Multifocal Entities in Patients with Papillary Thyroid Microcarcinoma" was retracted in 2024. Reasons: signs of a paper mill; suspected computer-generated content; unreliable results or conclusions; concerns about the data.

In the meantime, 9 cases in this study had a recurrence. Similar to the neck metastasis tendency in this study, group IV had the highest recurrence rate (3.6%), while the recurrence rate of group III was higher than that of group II (2.8% versus 1.2%). The difference was significant among the four groups (*p* = 0.021). Most probably due to the short follow-up period, we only had 9 patients with recurrence and could not draw any conclusion with statistical significance. However, a similar tendency for recurrence as that for CNM was indeed observed among the four groups. There were 10 cases with intraglandular dissemination in this study. Nine out of the 10 cases (90%) had unilateral multifocality, and only 3 cases (30%) had bilaterality, which was consistent with Bansal et al.'s finding that peritumoral dissemination is least seen in multifocal PTCs with different mutations, most of which appears as bilaterality [22]. Taken together, we concluded that (1) unilateral multifocality is a predictor for worse CNM than bilaterality in patients with PTMC, (2) unilateral multifocality and bilaterality could be two different kinds of multifocal entities, and (3) when unilateral multifocality and bilaterality coexisted in PTMCs, the patients have the highest risk of local metastasis and a higher propensity for local recurrence.

Patients with PTMC have a good overall prognosis. Based on this scenario, many researchers advocate more conservative and diversified treatment approaches [5, 29–32]. Under the circumstance that a prospective randomized control trial is not feasible, clinicians are interested in using scoring systems or criteria for stratification to accurately predict metastasis or recurrence risk and manage patients accordingly. In this study, age < 45 years, tumor size > 0.5 cm, male, and extrathyroidal invasion were all independent factors correlated with CNM in two separated multivariate analyses. Besides, tumor > 0.5 cm and CNM were correlated with LNM. All these results were consistent with previous reports [33–37], indicating that the patients in our study may not be different from other reports in mutation status and clinicopathological presentations, although areas and ethnic variations existed. Except the risk factors above, some studies suggest that PTMCs should also be classified as an incidental or nonincidental found microcarcinoma, as incidental PTMCs had significantly fewer aggressive tumor features and much better prognosis compared with nonincidental PTMCs [38–41]. In this study, no incidental PTMC was included, and all patients had evidence of malignance preoperatively.

The article "Unilateral Multifocality and Bilaterality Could Be Two Different Multifocal Entities in Patients with Papillary Thyroid Microcarcinoma" was retracted in 2024. Reasons: signs of a paper mill; suspected computer-generated content; unreliable results or conclusions; concerns about the data.

However, there are several limitations in the current study. Firstly, the median follow-up time was relatively shorter with few cases having a recurrence, leading to a limitation in investigating the correlation between recurrence and different clinicopathological factors. Secondly, lateral neck dissection was only performed on patients with macrometastasis. It is highly possible that many patients with occult LNM were missed, which would consequently affect the statistical analysis on the correlation between LNM and several risk factors (LNM was not significantly correlated with multifocality in this study). Thirdly, our hospital was not permitted to conduct radioiodine treatment with ^131^I, and we may not have complete records of the radioiodine treatment during follow-up, which could slightly affect the recurrence rate in this study, although only a limited number of patients were recommended to take radioiodine treatment.

In conclusion, unilateral multifocality and bilaterality could be two different kinds of multifocal entities in patients with PTMC. Patients with unilateral multifocality were more likely to have neck metastasis than those with bilaterality. When unilateral multifocality and bilaterality coexisted, patients with PTMC had the highest risk of CNM and possibly local recurrence compared with those with either risk factor alone.

## Figures and Tables

**Table 1:** Patient demographics.

Variables	Value
Total number	949
Age (years)	43.8 ± 11.3 (16-79)^a^
<45 years	490 (51.6)
≥45	459 (48.4)
Gender (M/F)	207/742
Tumor size (cm)	0.6 ± 0.2 (0.15-1)^a^
≤0.5	442 (46.6)
>0.5	507 (53.4)
Nodal involvement, n (%)	
Central neck metastasis	299 (31.5)
Lateral neck metastasis	44 (4.6)
Multifocality, *n* (%)	
Unilateral multifocality	155 (16.3)
Bilaterality	164 (17.3)
Capsular invasion	170 (17.9)
Perithyroidal invasion	21 (2.2)
Intraglandular dissemination	10 (1.1)
Hashimoto	179 (18.9)
Simple goiter	414 (43.6)
Thyroid surgery, *n* (%)	
Total thyroidectomy	169 (17.8)
Subtotal thyroidectomy	372 (39.2)
Lobectomy with isthmectomy	408 (43)
Central neck dissection, *n* (%)	
Unilateral	751 (79.1)
Bilateral	198 (20.9)
Modified lateral neck dissection	
Unilateral	61 (6.4)
Bilateral	3 (0.3)
Follow-up time (months)	32.2 (18-50)
Recurrence	9 (0.9)

^a^Mean ± standard deviation (range).

The article "Unilateral Multifocality and Bilaterality Could Be Two Different Multifocal Entities in Patients with Papillary Thyroid Microcarcinoma" was retracted in 2024. Reasons: signs of a paper mill; suspected computer-generated content; unreliable results or conclusions; concerns about the data.

**Table 2:** Risk factors of CNM.

	Univariate		Multivariate		
	OR (95% CI)	*p* value	*B* (SE)	*p* value	OR (95% CI)
Age (<45 vs. ≥45)	0.374 (0.280-0.499)	<0.001	-1.027	<0.001	0.358 (0.266-0.483)
Gender (female vs. male)	1.719 (1.249-2.365)	0.001	0.615	<0.001	1.849 (1.316-2.599)
Tumor size (≤0.5 vs. >0.5 cm)	2.356 (1.768-3.139)	<0.001	0.842	<0.001	2.320 (1.7213-3.129)
Unilateral multifocality	1.673 (1.174-2.384)	0.004	0.507	0.008	1.661 (1.142-2.416)
Bilaterality	1.405 (0.990-1.995)	0.056	/	/	/
Capsular invasion	1.534 (1.087-2.163)	0.014	/	/	/
Extrathyroidal invasion	3.648 (1.495-8.898)	0.002	1.023	0.033	2.783 (1.083-7.148)
Hashimoto	0.811 (0.566-1.162)	0.253	/	/	/
Simple goiter	0.780 (0.590-1.030)	0.08	/	/	/

**Table 3:** Risk factors of LNM.

	Univariate		Multivariate		
	OR (95% CI)	*p* value	*B* (SE)	*p* value	OR (95% CI)
Age (<45 vs. ≥45)	0.537 (0.284-1.015)	0.052	/	/	/
Gender (female vs. male)	1.921 (1.009-3.655)	0.043	/	/	/
Tumor size (≤0.5 vs. >0.5 cm)	4.146 (1.906-9.019)	<0.001	1.137	0.005	3.117 (1.413-6.879)
Unilateral multifocality	1.762 (0.870-3.566)	0.111	/	/	/
Bilaterality	1.244 (0.586-2.641)	0.569	/	/	/
Capsular invasion	1.773 (0.893-3.518)	0.097	/	/	/
Extrathyroidal invasion	2.221 (0.501-9.848)	0.254	/	/	/
Hashimoto	0.539 (0.209-1.387)	0.193	/	/	/
Simple goiter	1.440 (0.785-2.639)	0.236	/	/	/
CNM	5.668 (2.920-11.001)	<0.001	1.549	<0.001	4.708 (2.403-9.226)

**Table 4:** Clinicopathological factors between four groups classified by different multifocality status.

Variables	Groups				
	Group I (*n* = 713) (%)	Group II (*n* = 81) (%)	Group III (*n* = 72) (%)	Group IV (*n* = 83) (%)	*p* value
Age (≥45 vs. <45)	347/366 (48.7)	40/41 (49.4)	30/42 (41.7)	42/41 (50.6)	0.678
Gender (male vs. female)	157/556 (22)	15/66 (18.5)	21/51 (29.2)	14/69 (16.9)	0.261
Tumor size (>0.5 vs. ≤0.5)	360/353 (50.5)	56/25 (69.1)	38/34 (52.8)	53/30 (63.9)	0.003
Capsular invasion	125/588 (17.5)	15/66 (18.5)	13/59 (18.1)	17/66 (20.5)	0.927
Extrathyroidal invasion	17/696 (2.4)	2/79 (2.5)	0/72 (0)	2/81 (2.4)	0.622
Hashimoto	133/580 (18.7)	21/60 (25.9)	8/64 (11.1)	17/66 (20.5)	0.131
Simple goiter	328/385 (46)	19/62 (23.5)	41/31 (56.9)	26/57 (31.3)	<0.001
CNM	209/504 (29.3)	26/55 (32.1)	28/44 (38.9)	36/47 (43.4)	0.032
LNM	31/682 (4.3)	2/79 (2.5)	4/68 (5.6)	7/76 (8.4)	0.266
Recurrence	3/710 (0.4)	1/80 (1.2)	2/70 (2.8)	3/80 (3.6)	0.021

Group I: single lesion; group II: univocal bilaterality-single lesion in each lobe; group III: unilateral multifocality; group IV: unilateral multifocality and bilaterality coexist.

The article "Unilateral Multifocality and Bilaterality Could Be Two Different Multifocal Entities in Patients with Papillary Thyroid Microcarcinoma" was retracted in 2024. Reasons: signs of a paper mill; suspected computer-generated content; unreliable results or conclusions; concerns about the data.

**Table 5:** Predicting values of different multifocality status on neck metastasis.

	Univariate		Multivariate		
	OR (95% CI)	*p* value	*B* (SE)	*p* value	OR (95% CI)
CNM					
Age (<45 vs. ≥45)	0.374 (0.280-0.499)	<0.001	-1.033	<0.001	0.356 (0.264-0.480)
Gender (male vs. female)	1.719 (1.249-2.365)	0.001	0.632	<0.001	1.882 (1.339-2.645)
Tumor size (cm)	2.356 (1.768-3.139)	<0.001	0.833	<0.001	2.300 (1.705-3.102)
Capsular invasion	1.534 (1.087-2.163)	0.014	/	/	/
Extrathyroidal invasion	3.648 (1.495-8.898)	0.002	0.359	0.03	1.432 (1.036-1.979)
Univocal bilaterality^a^	1.030 (0.632-1.678)	0.905	/	/	/
Unilateral multifocality^b^	1.423 (0.867-2.334)	0.161	/	/	/
Bilaterality plus unilateral multifocality^c^	1.756 (1.111-2.775)	0.015	0.6	0.015	1.823 (1.122-2.961)
LNM					
Gender (female vs. male)	1.921 (1.009-3.655)	0.043	/	/	/
Tumor size (≤0.5 vs. >0.5 cm)	4.146 (1.906-9.019)	<0.001	1.137	0.005	3.117 (1.413-6.879)
Univocal bilaterality^a^	1.030 (0.632-1.678)	0.905	/	/	/
Unilateral multifocality^b^	1.423 (0.867-2.334)	0.161	/	/	/
Bilaterality plus unilateral multifocality^c^	1.756 (1.111-2.775)	0.015	/	/	/

Three kinds of multifocality forms were included in multivariate analysis along with other clinicopathological factors, which were significantly correlated with CNM or LNM in univariate analysis. ^a^Single lesion in each lobe. ^b^Unilateral multifocality. ^c^Unilateral multifocality and bilaterality coexist.

## Data Availability

The datasets generated during and/or analyzed during the current study are not publicly available, but are available from the corresponding author on reasonable request.
